# Proinflammatory Cytokines IL-6 and TNF-*α* Increased Telomerase Activity through NF-*κ*B/STAT1/STAT3 Activation, and Withaferin A Inhibited the Signaling in Colorectal Cancer Cells

This article has been retracted.

**DOI:** 10.1155/2017/5958429

**Published:** 2017-06-06

**Authors:** Seyung S. Chung, Yong Wu, Quincy Okobi, Debbie Adekoya, Mohammad Atefi, Orette Clarke, Pranabananda Dutta, Jaydutt V. Vadgama

**Affiliations:** ^1^Division of Cancer Research and Training, Department of Internal Medicine, Charles R. Drew University of Medicine and Science, 1731 East 120th street, Los Angeles, CA 90059, USA; ^2^Charles R. Drew University of Medicine and Science, 1731 East 120th street, Los Angeles, CA 90059, USA; ^3^David Geffen UCLA School of Medicine, Los Angeles, CA, USA; ^4^Jonsson Comprehensive Cancer Center, Los Angeles, CA, USA

## Abstract

There are increasing evidences of proinflammatory cytokine involvement in cancer development. Here, we found that two cytokines, IL-6 and TNF-*α*, activated colorectal cancer cells to be more invasive and stem-like. Combined treatment of IL-6 and TNF-*α* phosphorylated transcription factors STAT3 in a synergistic manner. STAT3, STAT1, and NF-*κ*B physically interacted upon the cytokine stimulation. STAT3 was bound to the promoter region of human telomerase reverse transcriptase (hTERT). IL-6 and TNF-*α* stimulation further enhanced STAT3 binding affinity. Stem cell marker Oct-4 was upregulated in colorectal cancer cells upon IL-6 and TNF-*α* stimulation. Withaferin A, an anti-inflammatory steroidal lactone, inhibited the IL-6- and TNF-*α*-induced cancer cell invasion and decreased colonosphere formation. Notably, withaferin A inhibited STAT3 phosphorylation and abolished the STAT3, STAT1, and NF-*κ*B interactions. Oct-4 expression was also downregulated by withaferin A inhibition. The binding of STAT3 to the hTERT promoter region and telomerase activity showed reduction with withaferin A treatments. Proinflammatory cytokine-induced cancer cell invasiveness is mediated by a STAT3-regulated mechanism in colorectal cancer cells. Our data suggest that withaferin A could be a promising anticancer agent that effectively inhibits the progression of colorectal cancer.

## 1. Introduction

Inflammation is one of the complex biological responses to the damages caused either by injury or microbial infection, where the immune system attempts to neutralize an injury. The role of inflammation in tumorigenesis is now widely accepted. In many cases, chronic inflammation in the microenvironment is essential for the initiation and progression of cancers. Although the molecular mechanisms by which the inflammation promotes cancer are explained, the molecular roles of inflammation in tumorigenesis, progression, and metastasis need to be better understood. Epidemiological evidence first points to a link between inflammation and a development of cancer [1]. It was reported that 15~20% of various cancer types have direct initiation cues from chronic inflammation in the same tissue or organ preceding the cancer development [2]. The risk of developing cancer from inflammation is often time-dependent on the type of cancer. Hepatitis or chronic inflammation caused by hepatitis B or C virus initiated hepatocellular carcinoma [3]. Chronic inflammatory diseases of small and large intestines, ulcerative colitis, and Crohn's disease provoked the development of colitis-related cancer [4].

Chronic inflammation is a risk factor for colorectal cancer development. Colorectal cancer is the second cancer-related mortality in the western world [5]. Over 50% of colorectal cancer patients eventually developed metastasis and recurrent colorectal cancer disease. There is an important association between colorectal cancer prognosis and cytokine levels in the serum of patients. When IL-6 (interleukin 6) and TNF-*α* (tumor necrosis factor *α*) coexpression is elevated, the prognosis of the patient is significantly poorer. It has been reported that IL-6 and TNF-*α* serum levels were elevated in colorectal cancer patients [6] and can be used as a prognosis factor [7]. Similarly, in breast cancer, the coexpression levels of IL-6 and TNF-*α* have been tightly associated with a negative prognosis [8]. Another study has shown that elevated serum levels of IL-6 were closely associated with the progress and prognosis of metastatic breast cancer [9]. Finally, patients with metastatic prostate cancer had significantly higher levels of serum IL-6 and TNF-*α* than primary cancer patients [10]. Taken together, these clinical reports implicate that IL-6 and TNF-*α* may function as a driver for cancer advancement, metastasis, and poor disease prognosis.

There is a notion that protumorigenic inflammation signaling pathways are subject to a feed-forward loop. We hypothesized that IL-6 and TNF-*α* contribute to the cancer initiation and progression by promoting cancer stemness and telomerase activity. To test this, we investigate the key transcription factors STAT3 (signal transducer and activator of transcription 3) and NF-*κ*B. STAT3 is a latent transcription factor that conveys the signals of growth factors and cytokines from the cellular membrane to nucleus onto its target genes [11]. STAT3 functions in a variety of physiological processes including embryonic development, immunity, and inflammation [12]. In addition, STAT3 transcriptionally activates the oncogenes, proliferative and angiogenesis-related genes in responding to the stimuli from outside, hence contributes to cancer progression [13]. NF-*κ*B (nuclear factor *κ*B) is a prominent transcription factor involved in immune response and inflammation. NF-*κ*B target genes are associated with the regulation of cell survival as well as apoptosis. Herein, we tried to identify the mechanisms of STAT3-NF-*κ*B-induced cancer cell activation. STAT3 activation resulted in the upregulation of stemness gene Oct-4. The activated transcription factors and increased telomerase were accordingly attributed to the cell invasiveness in the trans-well migration assay.

Natural compounds are major sources of current chemotherapeutic agents. Mounting evidence demonstrates the chemotherapeutic effects of natural compounds in preclinical and clinical studies. In an effort to find the novel natural compound to inhibit the cytokine signaling, we tried the withaferin A compound, which is abundant in Indian winter cherry. It is a steroidal lactone abundant in the plant *Withania somnifera* that has been used historically in oriental medicine, to treat inflammation and some neurological disorders [14, 15]. It has potent anti-inflammatory properties through the inhibition of Akt and NF-*κ*B signaling pathways [16, 17]. The antitumor, antimetastasis, and antiangiogenic activities of withaferin A have been reported from various cancer types [18]. The antiangiogenic property is linked to the degradation-enhancing modification of vimentin by withaferin A [19]. Recently, withaferin A showed the efficacious effects as an adjunct agent for chemotherapeutic agents, implicating to be well suited for an amplifier or supplementary agent alongside the conventional drug [20]. Withaferin A is an attractive anticancer agent based on the broad range of responses for the multiple cancers with a low toxicity. In this study, we investigated the molecular effects of withaferin A on cytokine-stimulated colorectal cancer cells. We have demonstrated that IL-6 and TNF-*α* cotreatments induce cancer cells to be more invasive and aggressive. We also report that withaferin A can inhibit the STAT3 activation, reduce the stem cell-like traits, and decrease the telomerase activity. These findings suggest the possible value of withaferin A in a novel therapy for the metastatic colorectal cancer.

## 2. Materials and Methods

### 2.1. Cell Culture and Reagents

DLD1 and HT-29 colorectal cancer cell lines were purchased from the American Type Culture Collection (ATCC, Manassas, VA, U.S.A.). Cancer cells were maintained in a monolayer culture in DMEM/F12 (Dulbecco's modified Eagle medium) with 10% fetal bovine serum, 1% L-glutamine, and 0.5% penicillin/streptomycin. Interleukin 6 was purchased from EMD Millipore (Temecula, CA, U.S.A. Catalog number: IL006). IL-6 was used at the concentration of 10 ng/ml to stimulate the cancer cells. We used the IL-6 concentration of 10 ng/ml according to the manufacturer's instruction. TNF-*α* was purchased from the R&D Systems (Minneapolis, MN; Catalog number: 210-TA-020). TNF-*α* was prepared as 100 *μ*g/ml stock solution. TNF-*α* concentration was decided based on the manufacturer's instructions. TNF-*α* was used at 25 ng/ml to activate cancer cells. Withaferin A was purchased from Sigma Aldrich company (Sigma Aldrich, St. Louis, MO; Catalog number: W4394). Withaferin A was prepared in 10 mM stock solution in methanol. The working concentration was 10 *μ*M for withaferin A in this study. Withaferin A concentration was decided based on the IC50 value from our dose-dependent cell growth study.

### 2.2. Western Blot Analyses

Monolayer cultures of respective cell lines at 80–90% confluence were lysed using 100 *μ*l of RIPA buffer (Thomas Scientific Inc. Swedesboro, NJ). Tris-glycine (Bio-Rad, Irvine, CA) gels were loaded with 100 *μ*g of total proteins. After electrophoresis, the gel was transferred to a nitrocellulose membrane for 1 hour.

The membrane was blocked for 30 min in 5% skim milk at room temperature. The membrane was briefly rinsed with 1xTTBS and incubated overnight with the respective primary antibodies at 4°C. Primary antibodies of STAT3, pSTAT3, NF-*κ*B, pNF-*κ*B, CD44, and Oct-4 were purchased from Cell Signaling Technology (Danvers, MA). Primary antibody for *β*-actin was purchased from the Santa Cruz Biotech (Santa Cruz, CA). After incubation with the secondary antibodies conjugated with horseradish peroxidase (HRP), the protein bands were developed with the chemiluminescent reagents.

### 2.3. Coimmunoprecipitation

Coimmunoprecipitation assay was performed as previously described [21]. Briefly, cells were washed once with PBS buffer and lysed in immunoprecipitation lysis buffer (Thomas Scientific Company). Antibodies to STAT3 (Cell signaling technology) were added to the cell lysates and incubated for one hour at 4°C. Protein A agaroses (Santa Cruz Biotechnology) were added to the cell lysates 20 *μ*l each, incubated for overnight at 4°C. After the immunoprecipitation, cell lysates were briefly spun and washed three times with 1X PBS buffer. Immunopellets were resuspended in 40 *μ*l of loading dye (Bio Rad) and run on a polyacrylamide gel electrophoresis. Immunoblots were probed for either NF-*κ*B or STAT1 proteins for interactions with STAT3 via western blot analyses.

### 2.4. CHIP (Chromatin Immunoprecipitation) Assay

Chromatin immunoprecipitation (ChIP) Assay Kit (Millipore, Catalog number: 17–295) was utilized to study STAT3 binding to hTERT promoter region. DLD1 or HT-29 cells were incubated with 1% formaldehyde for 20 minutes at 37°C. Cells were collected, lysed, sonicated, and incubated with 4 *μ*g of antibodies to STAT3 overnight. PCR was used to amplify DNA bound to the immunoprecipitated histones after reversing the histone-DNA cross-links. Primer sets were designed flanking the possible STAT3 binding regions. Primer sequences: *hTERT* promoter primer sequence 1, forward primer 5′- CCAAACCTGTGGACAGAACC-3′ and reverse primer 5′-AGACTGACTGCCTCCATCGT-3′ and *hTERT* promoter primer sequence 2, forward primer 5′-GGGGTGTCTTCTGGGTATCA-3′ and reverse primer 5′-AAGGGCTGTGTTTGTGAATTG-3′.

### 2.5. Telomerase Activity Assay

Telomerase activity assay was performed as previously described [22]. Briefly, cells were processed according to the manufacturer's protocol for the TeloTAGGG Telomerase PCR ELISA kit (Roche, Orange, CA. Catalog number: 11854666910). Briefly, cell pellets were thawed in lysis reagent, incubated on ice for 30 minutes, and centrifuged at 16,000*g* for 20 minutes at 4°C. Telomerase activity was immediately measured in the resultant supernatant using the telomeric repeat amplification protocol in which telomerase, if present in the cell lysate, adds telomeric repeats to the 3′ end of a biotin-labeled synthetic P1-TS primer. Samples were amplified by polymerase chain reaction (PCR), with P1-TS and P2 primers creating an elongated telomere. The PCR product was denatured and hybridized to a digoxigenin-labeled probe that detects telomeric repeats in a subsequent enzyme-linked immunosorbent assay (ELISA). Samples were considered positive for telomerase activity if the ELISA resulted in a background-corrected absorbance of ≥0.2 units. Telomerase assays were performed three times independently, and *p* values less than 0.05 were considered statistically significant.

### 2.6. Colonosphere Formation Assay

Colonosphere formation was examined as previously described [21]. Matrigel (BD, Cambridge, MA), 200 *μ*l was spread as a thick layer on wells of a 24-well plate and allowed to polymerize at 37°C for 15 minutes. 2 × 104 cancer cells grown in monolayer were trypsinized to single cells and plated on top of the precoated matrigel. Plates were incubated at 37°C to allow cells to fully settle down before media was replaced with appropriate culture media containing 5% matrigel. Cells were grown for 15 days; fresh growth media with matrigel was replenished every two days. Images of representative fields were taken.

### 2.7. Cell Invasion Assay

Cell invasion assay was performed as previously described [22]. Mouse fibroblasts (NIH-3T3) were used as a chemo-attractant and grown in a 24-well plate in 2 ml of DMEM/F12 media. Boyden chambers were prepared with 25 *μ*l of 1 : 6 diluted matrigel and allowed to incubate for 2 hours to solidify. Each chamber received the different treatments: methanol (vehicle) and withaferin A. After cell synchronization, an invasion was allowed to occur for 40 hours. The cells were then fixed with 0.5% glutaraldehyde and stained with 5% toluidine blue for cell counting.

### 2.8. Receptor Tyrosine Kinase Signaling Antibody Array Study

The receptor tyrosine kinase signaling antibody array kit was purchased from Cell Signaling Technology (Cell Signaling Technology, Beverly, MA; Catalog number: 7982). Each colorectal cancer cell line had stimulation by the IL-6 and TNF-*α* alone or in combination. Whole protein lysates were prepared using the provided lysis buffer from the kit. 100 *μ*l of each lysate was placed onto the membrane window of the antibody slide. The treated slide was incubated overnight at 4°C on an orbital shaker. The slide was then washed with 100 *μ*l 1X Array Wash Buffer and incubated on an orbital shaker for 5 minutes at room temperature. This washing procedure was repeated three more times. 75 *μ*l of 1X Detection Antibody Cocktail was added to each of the 8 wells, and the plate was covered with the provided sealing tape. It was incubated for 1 hour at room temperature on an orbital shaker. Next, three wash cycles were performed and the slide was incubated for 30 minutes with 75 *μ*l 1X HRP-linked Streptavidin. The slide was washed and treated with Lumi Glo and peroxide. We took the picture of the slides with a camera of gel documentation system (Bio-Rad, Gel Doc XRS) using Quantity One software.

### 2.9. Statistical Analysis

Student *t*-tests were used to evaluate the significance of changes in all combination treatment assays compared to controls. Data collected from each experiment was used to calculate the mean values and standard deviations (SD). Experiments were repeated three times independently. Differences were considered statistically significant if *p* < 0.05.

## 3. Results

### 3.1. IL-6 and TNF-*α* Cotreatments Activated STAT3 Synergistically Whereas Withaferin A Abolished the Activation

STAT3 and NF-*κ*B are key transcription factors activated in cells responding to inflammation. We first tested the effects of IL-6 and TNF-*α* cotreatments on the phosphorylation of STAT3 and NF-*κ*B (p65) in colorectal cancer cells. To this end, we performed the western blots for STAT3 and NF-*κ*B with the cancer cells treated with IL-6 alone, TNF-*α* alone, or IL-6 and TNF-*α* combined. As shown in Figure 1(a), IL-6 phosphorylated STAT3 whereas TNF-*α* did not phosphorylate it. When we cotreated cells with IL-6 and TNF-*α*, however, STAT3 phosphorylation levels were further elevated (Figure 1(a)). TNF-*α* may activate STAT3 indirectly as it enhances the IL-6 induction. We quantified the pSTAT3/STAT3 ratio using Image J software. IL-6 alone activated pSTAT3 to the 0.38 folds of total STAT3, but IL-6 and TNF-*α* cotreatments elevated the pSTAT3 level to 0.97 folds of STAT3 in DLD1 cell line (Figure 1(b)). Similarly, IL-6 alone increased pSTAT3 to 0.52 folds and combined IL-6 and TNF-*α* elevated pSTAT3 to 0.83 folds of STAT3 in HT-29. Our data suggest that IL-6 and TNF-*α* cotreatments activate STAT3. NF-*κ*B was phosphorylated by TNF-*α* alone or IL-6/TNF-*α* cotreatments. The NF-*κ*B activation was modest. Total STAT3 and NF-*κ*B levels were not changed upon IL-6 and TNF-*α* treatments.

Next, we tested if anti-inflammatory steroidal lactone withaferin A can deactivate pSTAT3 induced by IL-6 and TNF-*α* cotreatments. We hypothesized that withaferin A may exert anti-inflammatory effects through the downregulation of STAT3 phosphorylation. Indeed, withaferin A treatments inhibited the STAT3 phosphorylation in both DLD1 and HT-29 cancer cells (Figure 1(c)). NF-*κ*B phosphorylation levels were not changed upon withaferin A. Our results indicate that withaferin A may inhibit STAT3 activation selectively. With IL-6 and TNF-*α* stimulation, we wished to investigate Oct-4 expression levels. Tumor dedifferentiation is a well-known phenomenon, and it may involve in tumor progression [23]. Aberrant expression of Oct-4 is associated with abnormal tissue growth or tumorigenesis. Oct-4 is the most critical transcription factor since it can reprogram adult stem cells to iPS (induced pluripotent stem) cells as a single factor [24]. Oct-4 expression was also upregulated upon IL-6 and TNF-*α* cotreatments; however, in the presence of withaferin A, Oct-4 expression was downregulated (Figure 1(c)). IL-6 and TNF-*α* cotreatments activated STAT3 synergistically and upregulated Oct-4. Withaferin A abolished the STAT3 activation and prevented upregulation of Oct-4 expressions.

To examine time-dependent STAT3 and NF-*κ*B activation, we treated DLD1 cells with IL-6 and TNF-*α* on time points of 0, 6, 12, and 24 hours and examined the phosphorylation status. As shown in the Figure 1(d), both pSTAT3 and pNF-*κ*B were expressed from 6 hours and increased their expression levels to the 24 hour time points (Figure 1(d)).

### 3.2. STAT3 Physically Binds NF-*κ*B upon IL-6 and TNF-*α* Stimulation; However, Withaferin A Inhibits the STAT3-NF-*κ*B Interactions

Both STAT3 and NF-*κ*B are involved in gene regulation of inflammation and activated by IL-6 and TNF-*α*. We have previously shown that STAT3 and NF-*κ*B formed a complex and transcriptionally activated human telomerase reverse transcriptase in breast cancer lines of MDA-MB-231 and MCF7-HER2 [25]. We next wished to find out whether treatment with the combination of IL-6 and TNF-*α* can induce the interactions between STAT3 and NF-*κ*B in colorectal cancer cells. To uncover this, a coimmunoprecipitation assay was performed with cell extracts treated with IL-6 alone, TNF-*α* alone, or IL-6 and TNF-*α* combined. As shown in Figure 2, STAT3 was bound to NF-*κ*B with the IL-6 and TNF-*α* stimulations in both DLD1 and HT-29, respectively (Figures 2(a) and 2(c)). In DLD1 cells, IL-6 or TNF-*α* alone treatments were not sufficient to induce the STAT3-NF-*κ*B interactions (Figure 2(b)). Untreated cells also showed very weak binding to NF-*κ*B in HT-29 (Figure 2(d)). Our data suggest that activated STAT3 and NF-*κ*B physically interact upon IL-6 and TNF-*α* treatments.

Since withaferin A inhibited STAT3 activation, we tested whether the STAT3 interactions were abolished by withaferin A challenge. We performed the coimmunoprecipitation on the cell extracts treated with IL-6 and TNF-*α* with 10 *μ*M withaferin A this time. As withaferin A inhibited STAT3 phosphorylation, it also abolished the STAT3 interactions with NF-*κ*B in DLD1 and HT-29 (Figures 2(b) and 2(d)). Our results revealed the IL-6 and TNF-*α* cotreatments stimulated STAT3-NF-*κ*B complex, and withaferin A inhibited the STAT3-NF-*κ*B interactions.

### 3.3. STAT3 Binds to hTERT Promoter and Increases Telomerase Activity upon IL-6 and TNF-*α* Stimulation Whereas Withaferin A Inhibits STAT3 Binding and Decreases Telomerase

We next determined the STAT3 binding to hTERT (human telomerase reverse transcriptase) promoter region. It has been reported that STAT3 regulated the expression of hTERT in glioblastoma and primary cells [26]. We wished to determine whether transcription factor STAT3 was bound to hTERT promoter and further when stimulated by IL-6 and TNF-*α* if the binding was enhanced by these cytokines. To test this, we performed the Chip (chromatin immunoprecipitation) assay as described in Section 2. Consensus STAT3 binding sites (TTCNNNGAA) reside within the hTERT promoter. Chip assay was performed on the two putative STAT3-binding sites (Figure 3(a)). Cells were treated with IL-6, TNF-*α* alone, and combined. In DLD1 cells, we found that STAT3 was bound to the first STAT3 binding site located at −3308 base pair upstream hTERT open reading frame (Figure 3(b)). STAT3 binding affinity was approximately the same within the untreated control and TNF-*α* alone-treated samples. However, IL-6 and TNF-*α* cotreatments clearly enhanced STAT3 binding to the hTERT promoter region. These results suggest that transcription factor STAT3 is directly binding hTERT promoter and IL-6, and TNF-*α* cotreatments stimulate this binding. We investigated the telomerase activity upon activation and inhibition of STAT3 binding to hTERT promoter later.

STAT3 is phosphorylated in the cytoplasm, homodimerized with pSTAT3, and translocated into the nucleus to activate target genes. Since withaferin A inhibited STAT3 phosphorylation and its interactions with NF-*κ*B, we hypothesized that withaferin A may block the STAT3 binding to hTERT promoter. As shown in the Figure 3(c), 10 *μ*M withaferin A challenge blocked the STAT3 binding to the first STAT3 site within the hTERT promoter in our Chip assay (Figure 3(c)). This can be the effect of the reduced level of pSTAT3 in the presence of withaferin A since mainly pSTAT3 can translocate into nucleus and bind to the target gene promoters.

To measure the actual hTERT expression levels, we performed the western blots for hTERT with the IL-6-and TNF-*α*-treated cells and cytokine- and withaferin A-cotreated cells (Figure 3(d)). As shown in the figure, hTERT expression was upregulated with IL-6 and TNF-*α* stimulation whereas withaferin A cotreatment decreased hTERT expression. Our data show that STAT3 binding was enhanced by cytokine stimulation and translated into increased hTERT protein expression.

Finally, we examined the telomerase activity of colorectal cancer cells treated with IL-6, TNF-*α*, and withaferin A using TeloTAGGG Telomerase PCR ELISA kit as described in the methods section. Untreated DLD1 cells showed telomerase activity 2.67 (O.D. 450-O.D. 750). IL-6-treated cells and TNF-*α*-treated cells showed the telomerase activities of 2.68 and 2.72, respectively. Those activities are not statistically significant. However, when cells were cotreated with IL-6 and TNF-*α*, telomerase activity has been increasing to 3.04 (Figure 3(e)). This is 14% activity increase and out of standard deviation range. Withaferin A challenge clearly reduced the telomerase activity to 1.89. This is 29% decreased telomerase compared to the untreated control. To discern the telomerase difference more clearly, we reduced the cancer cell numbers from 2 × 105 to 1 × 104 and repeated the telomerase assay. Telomerase activity was increased from 0.58 to 0.77 with the IL-6 and TNF-*α* treatments whereas withaferin A (10 *μ*M) challenge decreased the activity to 0.255 (Figure 3(f)). Taken together, these results suggest that STAT3 directly bind to hTERT promoter, thereby regulating telomerase expressions; IL-6 and TNF-*α* cotreatments enhanced the STAT3 binding and increased effector protein telomerase activity. Anti-inflammatory withaferin A inhibited the STAT3 phosphorylation, blocked the binding to the hTERT promoter, and decreased telomerase activity.

### 3.4. Cotreatments with IL-6 and TNF-*α* Increased Cell Invasiveness Whereas Withaferin A Decreased both Colonosphere Formation and Trans-Well Invasion

As we found out the molecular mechanisms of STAT3 activation by cytokines of IL-6 and TNF-*α*, we next examined the cell-level invasiveness of colorectal cancer cells. To measure the cell invasiveness, we used two methods, colonosphere formation and trans-well invasion assays. For colonosphere formation, we created three-dimensional culture conditions by adding 5% matrigel to the 24-well plates. Cancer cells were seeded onto the wells with culture medium with or without IL-6 and TNF-*α*. Withaferin A treatment was done as a pretreatment in a 10 *μ*M withaferin A for 24 hours, and cells were seeded onto the wells. Formed colonospheres were counted after 14 days incubation. As shown in the Figure 4(a), untreated DLD1 cells formed ~29 spheres per wells whereas cytokine-treated cells showed increased spheres of ~71 (Figures 4(a) and 4(b)). However, withaferin A pretreatments almost abolished the sphere formation from the assay. Similarly, trans-well invasion assay showed ~30% of cell invasion with untreated ontrol while cytokine-treated cells showed 66% invasion. When cells were pretreated with withaferin A, the cell invasion has been decreased to 16% (Figures 4(c) and 4(d)). These data are consistent with the Chip assay and telomerase assay data in that cytokine-increased STAT3 binding and telomerase activity. On the contrary, withaferin A inhibited STAT3 activation decreased telomerase and cell invasiveness.

### 3.5. IL-6 Activated STAT3 and TNF-*α* Activated STAT1, STAT3, and STAT1 Heterodimerize upon IL-6 and TNF-*α* Cotreatments

Both IL-6 and TNF-*α* are pleiotropic cytokines stimulating more than one signaling pathways. We next investigated that which receptor tyrosine kinases were activated by IL-6 and TNF-*α* alone and in combination. To this end, we used the PathScan RTK Signaling Antibody Array Kit (Cell Signaling Technology) to screen the receptor tyrosine kinases. We were able to detect 28 receptor tyrosine kinases simultaneously using this array kit. We treated two cancer cell lines DLD1 and HT-29, then observed the receptor tyrosine kinase activation. When we treated with IL-6, STAT3 (Tyr 705) was phosphorylated whereas TNF-*α* treatment induced STAT1 (Tyr 701) phosphorylation in both DLD1 and HT-29 (Figures 5(a) and 5(b)). STAT1 is involved in upregulating genes due to a signal by either types I, II, or III interferons [27]. In response to stimulation, STAT1 forms homodimers or heterodimers with STAT3 that bind to the GAS (interferon-gamma-activated sequence) promoter element.

We next tested if STAT1 heterodimerize with STAT3, and furthermore, the interactions were enhanced by cytokine stimulation. To this end, we pulled down with STAT3 antibody and probed for STAT1 protein in the coimmunoprecipitation assay. As shown in the Figure 6(a), STAT1 heterodimerized with STAT3. When treated with IL-6 and TNF-*α*, the interaction was enhanced as the bound STAT1 protein amount was increased. We treated cells with chemotherapy agent 5-FU and withaferin A, then monitored the STAT3-STAT1 interactions. As shown in Figure 6(b), withaferin A abolished the STAT3-STAT1 interactions whereas 5-FU modestly reduced the interactions.

We have shown that STAT3 and NF-*κ*B physically bind from the previous coimmunoprecipitation study (Figure 2). We next tested if STAT1 also binds NF-*κ*B as STAT1 and STAT3 bind as well as STAT3 and NF-*κ*B bind. STAT1 pull-down assay showed that NF-*κ*B was bound to STAT1 (Figure 6(c)). When IL-6 and TNF-*α* were treated, the STAT1-NF-*κ*B interaction was also enhanced. We also treated 5-FU and withaferin A, then tested the STAT1-NF-*κ*B interactions. Withaferin A abolished the STAT1-NF-*κ*B interactions while 5-FU modestly decreased the binding. Our results suggest that IL-6 and TNF-*α* activate STAT3 and STAT1 on the receptor tyrosine kinase levels, then form the triplet complex with NF-*κ*B, subsequently induce cell invasiveness through the converged STAT3, STAT1, and NF-*κ*B regulations on the target genes in colorectal cancer cells.

## 4. Discussion

In this study, we found that STAT3 was synergistically activated by IL-6 and TNF-*α*. STAT3, STAT1, and NF-*κ*B formed triplet complexes with IL-6 and TNF-*α* stimulation, thereby increasing telomerase activity by binding hTERT promoter more tightly. Cell-level invasion assay revealed that cytokine treatments contributed to the cell invasiveness. An anti-inflammatory steroidal lactone withaferin A abolished the cancer stem cell traits and decreased telomerase activity significantly. Our data suggest the novel molecular mechanisms by which proinflammatory cytokines drive the colorectal tumorigenesis and a link between inflammation and cancer.

STAT3 and NF-*κ*B are transcription factors activated in the majority of cancers. They activate genes that control cell survival, proliferation, angiogenesis, invasiveness, and cytokine production [28, 29]. STAT3 and NF-*κ*B enhance resistance to apoptosis-based tumor surveillance of preneoplastic and malignant cells [30]. We found that combined treatments of IL-6 and TNF-*α* activate STAT3 in a synergistic manner, and promoted STAT3 and NF-*κ*B physically bind each other. With cytokine stimulation, STAT3 and NF-*κ*B formed a complex and activated their target genes, like hTERT. The IL-6-TNF*α* synergistic activation of STAT3 may result in the enhanced STAT3 activation on its target genes. Human TERT promoter region is likely one of the converging points of these activations elicited by the cytokines of IL-6 and TNF-*α*. In accordance, the telomerase activity was increased with the activation of STAT3 and NF-*κ*B. The next step of cytokine signaling characterization will be to monitor the changes in IL-6 and TNF-*α* production levels from the activated, telomerase-increased, and invasive cancer cells employing Elisa assays. If STAT3-NF-*κ*B signaling feed-forward loop working, the cytokine production possibly significantly increased in the invasive cells. More in vivo studies are warranted for the cytokine-stimulated tumorigenesis and withaferin A antitumor effects. The enhanced tumor formation with cytokines and tumor regression by withaferin A in an animal model is underway.

The cytokines, IL-6 and TNF-*α*, and transcription factors, STAT3 and NF-*κ*B, are critical for both inflammation and cancer, thus they can constitute a central signaling pathway that promotes inflammation and tumor growth concurrently. It has been shown that pharmacological interference on the cytokine signaling has decreased the tumorigenesis and cancer progression [31, 32]. Withaferin A has abolished the STAT3 activation in colorectal cancer cells. More importantly, withaferin A inhibited Oct-4, stem cell marker, expression in the cancer cells. Oct-4 is the most critical transcription factor for stemness, and aberrant Oct-4 expression is closely associated with abnormal tissue growth or tumorigenesis [33, 34]. There were multiple putative STAT3 binding sites in the Oct-4 promoter (Qiagen, Epi Tect ChIP qPCR data base). We also searched the current literature for the Oct-4 promoter binding proteins. The upstream signals that regulate Oct-4 expression and its gene circuitry are not well documented. More detailed Oct-4 gene regulation studies remain to be seen.

In addition, withaferin A decreased STAT3-NF-*κ*B interaction and significantly decreased telomerase activity. Presently, there is only one clinical trial going on with withaferin A at the University of Pittsburgh on Schizophrenia (Clinical Trial ID, NCT01793935). Based on our study and data from others, withaferin A is likely to be subject to new clinical trial for metastatic cancer. Considering withaferin A characteristics as a natural compound, it would be reasonable to use it as an amplifier or supplement for the standard chemotherapy agent for recurrent or metastatic cancers.

Our receptor tyrosine kinase array screen revealed that IL-6 induced STAT3 (Tyr 705) and TNF-*α* induced STAT1 (Tyr 701) activations. There has been a report that a low STAT1 and high STAT3 ratio showed faster tumor growth in a xenograft [35]. Accordingly, these results reflected the similar clinical outcomes from the colorectal cancer patients. When STAT1 is low and STAT3 is high, the prognosis was poor. It was proposed that the ratio of STAT1 to STAT3 expression was a key determinant of colorectal cancer progression and that STAT1 counteracts protumorigenic STAT3 signaling. Our data indicate that TNF-*α* elicits STAT1 pathway and IL-6 activates STAT3 pathway in terms of receptor tyrosine kinase levels. STAT3 and STAT1 activation and dimerization can be a regulation mechanism for IL-6 and TNF-*α* signaling. One step further, NF-*κ*B also complexed with STAT3 and STAT1 and contributed to the target gene activation. One similar study to our work has been reported from the breast cancer area. Snyder and associates have shown that STAT3-NF-*κ*B complex was necessary for the expression of fascin in metastatic breast cancer cells in response to IL-6 and TNF-*α* [36]. In there, they showed that treatment of IL-6 and TNF-*α* led to the formation of STAT3 and NF-*κ*B, binding to the fascin promoter region. STAT3-NF-*κ*B complex was necessary for the fascin expression and migration of breast cells. More characterization of the STAT3-STAT1 dual regulation on the cancer stemness and telomerase studies remains to be seen.

## Figures and Tables

**Figure 1:** STAT3 was activated by IL-6 and TNF-*α* treatments whereas inhibited by withaferin A in human colorectal cancer cells. (a) Western blot analysis of DLD1 and HT-29 for pSTAT3, total STAT3, pNF-*κ*B, and total NF-*κ*B. Cells were treated with IL-6 (10 ng/ml) and TNF-*α* (25 ng/ml) alone and in combination for 24 hours, then subjected to protein analysis for pSTAT3, total STAT3, pNF-*κ*B, and total NF-*κ*B. (b) A quantitative graph of pSTAT3: STAT3 ratio was presented from DLD1 and HT-29 (^∗^*p* < 0.05, ^∗∗^*p* < 0.001). (c) Western blot analysis of DLD1 and HT-29 for pSTAT3, pNF-*κ*B, and Oct-4. Cells were treated with either IL-6 (10 ng/ml) and TNF-*α* (25 ng/ml) alone or in combination for 24 hours. Withaferin A was treated at 10 *μ*M concentrations for 24 hours as indicated. (d) STAT3 and NF-*κ*B phosphorylation was measured with IL-6 and TNF-*α* stimulation on a time course. DLD1 cells were treated with combined IL-6 and TNF-*α* and monitored the phosphorylation status on different time points of 0, 6, 12, and 24 hours.

**Figure 2:** STAT3 and NF-*κ*B bind upon IL-6 and TNF-*α* treatments in colorectal cancer cell lines DLD and HT-29. (a) Immunoprecipitation with STAT3 antibody revealed that NF-*κ*B was bound to STAT3 in DLD1 cell line. STAT3 pull-down was performed in the presence of IL-6 (10 ng/ml) and TNF-*α* (25 ng/ml). (b) In the presence of withaferin A (10 *μ*M), pull-down assay with STAT3 antibody showed that STAT3 interaction with NF-*κ*B was abolished in DLD1 cell line. (c) Immunoprecipitation with STAT3 antibody showed the interactions with NF-*κ*B in HT-29 cell line. (d) With the withaferin A challenge (10 *μ*M), STAT3 and NF-*κ*B interactions were abolished in HT-29.

**Figure 3:** STAT3 binds hTERT promoter region. There are two STAT3 binding sites located in the promoter region of hTERT. Primer sets were designed flanking the putative STAT3-binding sites 1 and 2. Chip assay was performed with the primers. (a) Diagram of hTERT promoter with location of consensus STAT3-binding sites 1 and 2 indicated. (b) Chip assay was performed with the DLD1 lysates using anti-STAT3 antibody. Cells were pretreated with IL-6 and TNF-*α* alone or in combination. (c) Chip assay was performed with DLD1 cells stimulated with IL-6 and TNF-*α*, and DLD1 cells cotreated with IL-6, TNF-*α*, and withaferin A. (d) Western blot of hTERT proteins. DLD1 cells were treated with IL-6 and TNF-*α* and cotreated with IL-6, TNF-*α*, and withaferin A and monitored for the hTERT expression levels. (e) TRAP-PCR-ELISA assay for telomerase activity. DLD1 cells of 2 × 105 were treated with IL-6 (10 ng/ml) for 24 h, TNF-*α* (25 ng/ml) for 24 h alone, and in combination. Withaferin A (10 *μ*M) was treated with the cytokines and applied to TRAP-PCR-ELISA assay to monitor telomerase assay. Telomerase activities were measured three times independently. All of the data are presented as mean ± SD (*n* = 3 in each group). ^∗^*p* < 0.05, ^∗∗^*p* < 0.01 versus untreated control. (f) Less amount of cells, 1 × 104, was treated with IL-6 and TNF-*α* alone and in combination. We decreased the cell amounts to discern cytokine and withaferin A effects on telomerase more clearly. ^∗^*p* < 0.05, ^∗∗^*p* < 0.01 versus untreated control.

**Figure 4:** IL-6 and TNF-*α* cotreatments increased colonosphere formation and cell invasion whereas withaferin A decreased the sphere formation and cell invasiveness. (a) Colonosphere formation assay. DLD1 cells were cotreated with IL-6 and TNF-*α* for 24 hours, then subjected to the three-dimensional culture condition. Withaferin A (10 *μ*M) was pretreated with IL-6 and TNF-*α*, then applied to three-dimensional culture. Representative images were taken after 7 days. Scale bar represents 50 *μ*m in length. (b) Quantitative representation of colonospheres formed in IL-6 and TNF-*α* cotreatments in the absence and presence of withaferin A. ^∗^*p* < 0.05, ^∗∗^*p* < 0.01 versus untreated control. (c) Boyden chamber assay. Cell invasiveness was examined by employing Boyden chamber assay. Human colorectal cancer DLD1 cells were subjected to Boyden chamber cell invasion assay. Cells were treated with IL-6 and TNF-*α* in the absence or presence of withaferin A. Assays were done for 48 hours. Representative images were taken. Scale bar represents 50 *μ*m in length. (d) The cell invasion assay was quantitatively measured in graphic representation. ^∗^*p* < 0.05, ^∗∗^*p* < 0.01 versus untreated control.

**Figure 5:** IL-6 activated STAT3 (Tyr 705) and TNF-*α* activated STAT1 (Tyr 701) in human colorectal cancer cells. We investigated the receptor tyrosine kinase phosphorylation with IL-6 and TNF-*α* treatments in DLD1 and HT-29. (a) When DLD1 cell was treated with IL-6 (10 ng/ml), STAT3 was activated. TNF-*α* treatment activated STAT1 (Tyr 701). IL-6 and TNF-*α* cotreatments activated both STAT1 and STAT3. (b) HT-29 was treated with TNF-*α* and IL-6. TNF-*α* treatments activated STAT1 (Tyr 701). IL-6 treatment activated STAT3 (Tyr 705).

**Figure 6:** STAT3 dimerize with STAT1 and STAT1 dimerize with NF-*κ*B. Withaferin A abolished the protein-protein interactions. (a) STAT1 was heterodimerized with STAT3 from the pull-down assay with an STAT3 antibody. The binding affinity was increased upon IL-6 and TNF-*α* cotreatments. (b) Withaferin A (10 *μ*M) treatment has abolished the STAT3-STAT1 interactions. (c) Coimmunoprecipitation with STAT1 antibody revealed that STAT1 was bound to NF-*κ*B. STAT1-NF-*κ*B interaction was enhanced by the IL-6 and TNF-*α* stimulation. (d) These interactions were also abolished by withaferin A (10 *μ*M) treatment.
